# Prevalence and Risk Factors for Allergic Rhinitis in China: A Systematic Review and Meta-Analysis

**DOI:** 10.1155/2022/7165627

**Published:** 2022-09-23

**Authors:** Kaiyun Pang, Guodong Li, Mouhan Li, Lan Zhang, Qinwei Fu, Kepu Liu, Wei Zheng, Zhiqiao Wang, Juan Zhong, Lijin Lu, Peijia Li, Yucan Zhou, Wanling Zhang, Qinxiu Zhang

**Affiliations:** ^1^Department of Otolaryngology, Hospital of Chengdu University of Traditional Chinese Medicine, Chengdu University of Traditional Chinese Medicine, Chengdu 610075, China; ^2^Department of Otolaryngology, Kaifeng Hospital of Traditional Chinese Medicine, Kaifeng 475000, China; ^3^Department of Otolaryngology, Shanxi Provincial People's Hospital-The Fifth Clinical Medical College of Shanxi Medical University, Taiyuan 030000, China; ^4^Department of Radiology, Kaifeng Children's Hospital, Kaifeng 475000, China; ^5^Department of Otolaryngology, School of Medical and Life Sciences & Reproductive & Women-Children Hospital, Chengdu University of Traditional Chinese Medicine, Chengdu 611137, China

## Abstract

The prevalence of allergic rhinitis (AR) has increased tremendously in the recent year in China. Evidence-based medicine to objectively evaluate the prevalence and risk factors for AR in China is urgently required. Toward this, we systematically searched four English and four Chinese databases to identify the literature on the same, from the year of website establishment until November 2021. A total of 51 studies were evaluated, and data were obtained through Stata 16 analysis. Overall pooled risk factors for adult AR were smoking (odds ratio [OR] = 1.89, 95% confidence interval [CI]: 1.25, 2.87), asthma (OR = 3.30, 95% CI: 1.48, 7.39), a family history of AR (OR = 3.17, 95% CI: 2.31, 4.34), a family history of asthma (OR = 3.99, 95% CI: 2.58, 6.16), drug allergy (OR = 1.62, 95% CI: 1.38, 1.89), food allergy (OR = 2.29, 95% CI: 1.39, 3.78), pollen allergy history (OR = 2.41, 95% CI: 1.67, 3.46), antibiotic use (OR = 2.08, 95% CI: 1.28, 3.36), occupational dust exposure (OR = 2.05, 95% CI: 1.70, 2.47), home renovation (OR = 1.73, 95% CI: 0.99, 3.02), and middle school education (OR = 1.99, 95% CI: 1.29, 3.06). Overall pooled risk factors for AR in children were passive smoking (OR = 1.70, 95% CI: 1.02, 2.82), asthma (OR = 3.26, 95% CI: 2.42, 4.39), a family history of AR (OR = 2.59, 95% CI: 2.07, 3.24), a family history of allergy (OR = 4.84, 95% CI: 3.22, 7.26), a history of allergic diseases (OR = 2.11, 95% CI: 1.52, 2.94), eczema(OR = 2.29, 95% CI: 1.36, 3.85), owning pets (OR = 1.56, 95% CI: 1.37, 1.77), eating seafood (OR = 1.30, 95% CI: 1.10, 1.55), boys (OR = 1.58, 95% CI: 1.43, 1.74), and breastfeeding (OR = 0.82, 95% CI: 0.55, 1.22). The results of our meta-analysis showed that the prevalence of allergy rhinitis was 19% (95% CI 14–25) among adults and 22% (95% CI 17–27) among children, with boys showing a higher prevalence than girls. The development of AR in China is associated with several factors, including allergic diseases (eczema, asthma, pollen allergy, and food allergy), a family history of allergy (AR, asthma, and other allergies), and dwelling and working environment (smoking or passive smoking, occupational dust exposure, and owning pets); conversely, breastfeeding can reduce the risk.

## 1. Introduction

Allergic rhinitis (AR) is induced by immunoglobulin E-mediated nasal infection leading to a series of nasal mucosa dysfunction of associated symptoms and concurrently affecting quality of life; the AR incidence has increased globally over time [1, 2]. The AR incidence ranges from 12.8% in Spain to 65.9% in New Zealand, more than 50% in some high-income countries, inversely in middle-income countries, and comparatively low in low-income countries [1, 3]. With the demographic transition, AR morbidity has shown a tremendous growth in its epidemiology and imposes a heavy socioeconomic burden on patients [4]. In Asia, the socioeconomic burden of AR and urticaria ranges from $ 30.7 to $105.4 billion, of which the Korean AR expense constitutes almost $272.92 million in direct medical care [5, 6].

With the acceleration of industrialization and urbanization, respiratory problems have increased and become a focus of concern in China [7]. Cross-sectional population-based studies in multiple Chinese cities demonstrated that the adult AR prevalence ranged from 9.6 to 23.9% and a mean of 9.8% in children in different parts of northern and southern China [8, 9]. In recent years, this disease has shown increased prevalence. The epidemiological data with respect to the prevalence of AR vary considerably in different Chinese cities. Indeed, seeking evidence-based medicine to objectively evaluate the prevalence of AR and anecdotal evidence in China is urgently required.

Although the etiology of AR is not obvious, fungal spores, climate factors, indoor environment, ambient air pollution, and inherent characteristics may attribute to its occurrence [10–12]. Examination of trends in the prevalence of AR is imperative for monitoring this health priority. Effective avoidance and identification of risk factors are warranted that contribute to the treatment and precautions against AR. However, which risk factors are important for AR in China? Current literature evidence shows uneven quality and inconclusive data. This review discusses the AR epidemiology and risk factors in China by collecting all the research data using evidence-based medicinal methods to identify significant risk factors for the systematic prevention and control of AR.

## 2. Materials and Methods

### 2.1. Literature Search Methods

We searched the electronic databases such as PubMed, EMBASE, the Cochrane Library, Web of Science, China National Knowledge Infrastructure China Biology Medicine Disc, WANFANG database, and Chongqing VIP database from the year of website establishment until November 2021. The systematic review was conducted according to the observational study methodology of Cochrane recommendations and registered at PROSPERO under the registration number CRD42022299105. The search process was conducted using the terms: “Rhinitis, Allergic,” “Epidemiology,” and “Prevalence,” and the following keywords: (“rhinitis, allergic” OR “allergic rhinitides” OR “allergic rhinitis”) AND (“Epidemiology” OR “Epidemiology” OR “social epidemiology” OR “social epidemiologies” OR “Prevalence” OR “period prevalence” OR “period prevalences” OR “prevalence period” OR “point prevalence” OR “point prevalences” OR “prevalence point” OR “Morbidity” OR “incidence” OR “effect”) AND “China.”

### 2.2. Inclusion and Exclusion Criteria

The inclusion criteria were as follows: (1) all investigative studies or reports with a diagnosis of AR, (2) integrity and reproducible originality of data, (3) risk factors studies that calculated outcome with corresponding 95% confidence interval (CI) and adjusted odds ratio (including smoking and allergy history), and (4) language restricted to Chinese and English.

The exclusion criteria were as follows: (1) duplicate, incomplete, incorrect, or unusable data, (2) comments, conferences, reports, and reviews, (3) non-up-to-date data and comprehensive data in the same region, (4) vague sample source, inclusion, and exclusion criteria, (5) special groups, such as officers, pilots, and nurses, and (6) the literature quality score of *C*.

### 2.3. Data Extract and Literature Quality Assessment

The parameters were extracted independently by two persons who conducted preliminary screening and cross-checking of data for quality control. When the results of both parties were inconsistent, a third party stepped in to help work out the problem. The extracted content of literature information included author, publication year, region, age, incidence and corresponding research results, case load, and risk factors. Depending on the methods of risk assessment criteria for cross-sectional study bias, outcome, comparability, and selection of study subjects, the study quality was evaluated independently by using the Combie checklist for the cross-sectional study. The seven terms are reassigned one point for each item, with a response of “yes” scoring 1 point, “no” scoring 0 points, and “not clear” scoring 0.5 points. *A* is assigned a score of 6–7, *B* is assigned 4.0–5.5, and *C* is under 4 score.

### 2.4. Statistical Methods

The data processing was conducted using the software Endnote *X*9 screening of the qualified literature, Excel 2019 extracting relational data, and Stata 16 analysis data. Heterogeneity between study results was determined by *I*^2^ when *I*^2^ >50% meant greater heterogeneity among the studies, using the random effects model. Risk factors sensitivity analysis was conducted using combined OR and 95% CI and compared using the fixed effects model and the random effects model to test for the results' robustness. Egger's test was used to evaluate publication bias wherein the conclusion was considered biased if *p* < 0.05.

## 3. Results

Overall, 10,701 studies were initially identified from the databases according to the inclusion criteria. After excluding ineligible studies meeting the exclusion criteria such as duplicates, incomplete, incorrect, or unusable data, 51 studies were finally included in the review, and the flow diagram of the study design is shown in Figure 1. Detailed characteristics of the studies, which included 12 adult studies [13–24] and 23 children's studies [15, 18–20, 22, 25–42], are shown in Tables 1 and 2. Seventeen studies [13, 15, 16, 18, 19, 24, 43–52] reporting adult risk factors and 16 studies [9, 19, 28, 32, 35, 38, 39, 53–61] reporting children's risk factors constituted the final included studies on AR.

### 3.1. Sensitivity Analysis for Overall Prevalence of AR

After Stata verification, the overall pooled prevalence of AR in adults was 19% (95% CI 14–25) (Figure 2), and the sensitivity analysis is shown in Figure 3. The overall pooled prevalence of AR in children was 22% (95% CI 17–27) (Figure 4), and the sensitivity analysis is shown in Figure 5. The sensitivity analysis was removed when any one study in Stata soft showed that the results have no significant publication bias and stability in adults, same as in children.

### 3.2. Risk Factors

#### 3.2.1. Overall Adult Risk Factor Outcomes

Among the risk factors for adult AR included in the literature, a family history of asthma, drug allergy, pollen allergy history, and occupational dust exposure were selected for the fixed effect analysis method to evaluate on the basis of *I*^2^ <50% and combined effect size. Smoking, asthma, food allergy, antibiotic use, home renovation, and middle school education were chosen for the random effect analysis method to calculate on the basis of I^2^ >50% and combined effect size. The meta-analysis results revealed that the combined effect sizes of all other risk factors were statistically significant, except for the association between home decoration and adult AR (Figure 6).

#### 3.2.2. Overall Children's Risk Factor Outcomes

Among the risk factors for children with AR, passive smoking, asthma, a family history of AR, eczema, male sex, and breastfeeding were selected for the random effects model due to heterogeneity on the basis of *I*^2^ >50% and combined effect size. A family history of allergy, a history of allergic diseases, owning pets, and eating seafood were chosen for the fixed effects model on account of heterogeneity *I*^2^ <50% and combined effect size. Breastfeeding was a protective factor (95% CI 0.82 (0.55, 1.22), *p*=0.326), and a family history of allergy was the primary risk factor (95% CI 4.84 (3.22, 7.26), *p* < 0.001) for AR in children (Figure 7).

#### 3.2.3. Sensitivity Analysis and Egger's Test

A statistical comparison of the fixed effects and random effects models of risk factors showed consistent and reliable results. Egger's test of risk factors for children indicated a publication bias for a history of allergic diseases and eating seafood (*p* < 0.05). Egger's test of risk factors for adults showed no significant publication bias (Figures 8 and 9).

### 3.3. Detailed Risk Factor Results

#### 3.3.1. Smoking and Passive Smoking

Six studies on adult smoking [13, 15, 19, 43–45] and seven studies on passive smoking in children [32, 54–59] used regression analysis of multiple factors of AR outcomes. Two studies [32, 54] found no significant correlation between passive smoking and AR in children; however, the overall pooled analysis showed an association between smoking and adult AR. The statistical analysis for an association between smoking in adults and passive smoking in children and AR (OR_adult_ 1.89, 95% CI [1.25, 2.87] and OR_children_ 1.70, 95% CI [1.02, 2.82]) showed that smoking was a significant risk factor for AR.

#### 3.3.2. Asthma

Four studies [15, 16, 18, 46] on the asthma-related comorbidity in adults and six studies [9, 39, 56–59] on the same in children used regression analysis of multiple factors of AR outcomes. Asthma was associated with AR in adults and children (OR_adult_ 3.30, 95% CI [1.48, 7.39] and OR_children_ 3.26, 95% CI [2.42, 4.39]); thus, asthma was remarkably correlated with AR.

#### 3.3.3. Eczema

Three studies [9, 39, 54] that examined the association between eczema and AR found its unfavorable association with AR in children. The overall pooled risk factor of eczema was OR 2.29, 95% CI (1.36, 3.85).

#### 3.3.4. Family History of AR

Ten studies [16, 18, 19, 43–48] in adults and eight studies [19, 28, 39, 55–59] in children examined the relationship between a family history of AR and AR showed that it was a significant risk factor. The overall pooled family history of AR was OR 3.17, 95% CI (2.31, 4.34) in adults and OR 2.59, 95% CI (2.07, 3.24) in children.

#### 3.3.5. Family History of Asthma

Three studies [16, 43, 46] reported the association between a family history of asthma and AR in adults. We found a significant correlation between a family history of asthma and AR overall, as shown by OR 3.99, 95% CI (2.58, 6.16) in adults.

#### 3.3.6. Family History of Allergy

Four studies [35, 38, 54, 60] examined a family history of allergy as a risk factor for AR in children. We found a significant association between a family history of allergy and AR overall, as shown by OR 4.84, 95% CI (3.22, 7.26) in children.

#### 3.3.7. History of Allergic Diseases

Four studies [55, 56, 58, 59] reported a history of allergic diseases as a risk factor for AR in children. We found that a history of allergic diseases was a significant risk factor for AR, as shown by OR 2.11, 95% CI (1.52, 2.94) in children.

#### 3.3.8. Drug Allergy

Three studies [15, 19, 46] examined the association between drug allergy and AR in adults, and the analysis results showed that drug allergy was a significant risk factor for AR, as shown by OR 1.62, 95% CI (1.38, 1.89) in adults.

#### 3.3.9. Food Allergy

Four studies [15, 19, 45, 46] reported food allergy as a risk factor for AR in adults. Our analysis showed a significant association between food allergy and AR, which is shown by OR 2.29, 95% CI (1.39, 3.78) in adults.

#### 3.3.10. Pollen Allergy History

Three studies [18, 45, 49] examined the association between pollen allergy history and AR in adults. Of these, one study [45] found no significant correlation, but the overall analysis showed OR 2.41, 95% CI (1.67, 3.46) that indicated pollen allergy history as a significant risk factor for AR in adults.

#### 3.3.11. Antibiotic Use

Three studies [15, 19, 43] examined the association between antibiotic use and AR diseases and found it to be unfavorably associated with AR in adults. The overall pooled antibiotic use showed OR 2.08, 95% CI (1.28, 3.36).

#### 3.3.12. Owning Pets

Eight studies [38, 39, 54–56, 58, 59, 61] examined the association between owning pets and AR in children. One study [54] found no significant association, but the overall pooled pet ownership was OR 1.56, 95% CI (1.37, 1.77),which indicated that pets were significant risk factors for AR in children.

#### 3.3.13. Occupational Dust Exposure

Three studies [18, 49, 50] reported occupational dust exposure as a risk factor for AR in adults. We found a significant correlation between occupational dust exposure and AR (OR 2.05, 95% CI (1.70, 2.47)) in adults.

#### 3.3.14. Eating Seafood

Three studies [39, 55, 59] that examined the association between eating seafood and AR diseases found it to have an unfavorable association with AR in children. The overall pooled risk factor of eating seafood was OR 1.30, 95% CI (1.10, 1.55) in children.

#### 3.3.15. Home Renovation

Three studies [15, 48, 51] examined the relation between home renovation and AR in adults. Our analysis results indicated no significant association between home renovation and AR (*p*=0.056).

#### 3.3.16. Boys

Four studies [9, 32, 35, 53] reported boys as a risk factor for AR in children, and our analysis supported this conclusion. The overall pooled risk factor of boys was OR 1.58, 95% CI (1.43, 1.74) in children.

#### 3.3.17. Middle School Education

Five studies [13, 19, 24, 46, 52] examined the association between the level of education and AR. Our analysis showed a significant correlation between education and AR, indicating that individuals with secondary education were more likely to experience AR, OR 1.99, 95% CI (1.29, 3.06).

#### 3.3.18. Breastfeeding

Seven studies [9, 38, 53, 55, 56, 58, 59] reported the association between breastfeeding and AR. We found breastfeeding is stated to be a protective factor between breastfeeding and AR with OR 0.82, 95% CI (0.55, 1.22), *p*=0.326.

## 4. Discussion

The main purpose of this study was an assessment of the prevalence of AR and risk factors for AR among adults and children in China. The results of our meta-analysis showed that the prevalence of AR was 19% among adults and 22% among children in China. Regional differences have been observed in the prevalence of AR in China, with the lowest rate in the southern areas and the highest in northern China and high morbidity rates in cities with developed economies and industries, which is consistent with the incidence of AR in Europe [62, 63]. Comparing sex-related differences in the prevalence of AR in children, boys showed a higher prevalence than girls [9, 32, 35, 53], revealing that sex is also a definite risk factor for AR. Sex as a risk factor is a controversial factor in adults, as previous studies showed conflicting results including no sex-specific prevalence difference, male sex not significantly associated with allergic rhinitis and female sex being more susceptible [64–67]. There are also substantial gaps in the AR literature regarding whether sex is a risk factor in adults, which requires further confirmation.

AR, as a respiratory inflammatory disease, constitutes a complex immunological response in nasal mucous membranes and is closely related to environmental exposure. Allergies or a history of allergies and their incidence were determined by specific risk factors and intricate interplay of environmental exposures and genetic. Epigenetics have highlighted an association between subsequent risk and environmental exposures for AR and deserve further exploration in the pathogenesis of AR; these include a study of miRNA levels, histone acetylation, and alteration of DNA methylation [68, 69]. Murine studies have shown that epigenetically modified dendritic cells transmit the allergic risk from mothers to offspring [70]. Another study demonstrated that maternal and paternal allergy were important risk factors for AR in offspring [71, 72]. Consistent with the findings of this study, the current study also found that a history of allergies was intensely relevant to the development of AR. Therefore, the high-risk group with a family history of allergies would need to be monitored with a regular physical examination and early intervention to prevent AR.

Allergic diseases, AR, eczema, and asthma have close relationship due to overlapping genetic characteristics [68]. Our results support the findings, as we observed that allergic rhinitis, which is an allergic disease, was a significant risk factor for AR as it involves specific susceptibility loci associated with epithelial barrier functions, regulatory *T* cells, and interleukin-1 family signaling in pathogenic diseases, confirming an essential role in lymphocyte-mediated immunity [70, 73, 74]. Therefore, preventing eczema and asthma to a certain extent by active prevention and treatment may decrease the occurrence of AR. Allergic diseases may induce AR by food allergy, which is considered a manifestation of immune dysfunction [75, 76]. We found that food allergy and drug allergy were risk factors for AR; thus, proactively managing allergens is crucial to avoid exposure to allergens.

Our results indicated that home renovation, occupational dust exposure, owning pets, and pollen allergy played a role in the development of AR, as well as some strong environmental factors, which ranged from personal living habits to many different exposures in both external environment and home. Although most of the factors studied were risk factors for AR, home renovation indicated no significant association in adults. Therefore, for high-risk patients, it is highly recommended that there should be no pets or plants, hygiene should be maintained, and indoor ventilation should be cleaned regularly to minimize the exposure to allergens.

Breastfeeding reduces the risk of AR disease because the breast milk constituent, including long chain fatty acids, cytokines, and immunoglobulin *A*, stimulates the immune response and modify the balance between the anti-inflammatory and proinflammatory status [77]. The findings of this review revealed that breastfeeding as a protective factor influenced the immune system.

Due to the biases in investigative studies, the conclusion of the review should contain consideration for different geographical regions and observation over time. The limitations of this study were as follows: (1) Geographic and demographic biases may exist. (2) Egger's test found that two factors, a history of allergic diseases and eating seafood, had a certain publication bias; therefore, these results need to be confirmed by further research, and (3) some risk factors could not be analyzed because of the limited available literature.

## 5. Conclusions

In summary, the prevalence of AR was related to a variety of factors. Therefore, further studies in different geographical regions of China should be conducted with a focus on different risk factors. These studies may provide more information about the disorder and medical assistance using strategies to reduce the risk of AR among Chinese adults and children.

## Figures and Tables

**Figure 1:** Flow diagram of the studies included in the meta-analysis.

**Figure 2:** The forest plot of overall prevalence of allergic rhinitis in adults.

**Figure 3:** The sensitivity analysis of overall prevalence of allergic rhinitis in adults.

**Figure 4:** The forest plot of overall prevalence of allergic rhinitis in children.

**Figure 5:** The sensitivity analysis of overall prevalence of allergic rhinitis in children.

**Figure 6:** Heterogeneity test and meta-analysis results of adult risk factors.

**Figure 7:** Heterogeneity test and meta-analysis results of children risk factors.

**Figure 8:** Adult sensitivity analysis and Egger's test.

**Figure 9:** Children sensitivity analysis and Egger's test.

**Table 1:** Characteristics of the adult morbidity studies included in the meta-analysis.

First author (year)	Geographical zone	Survey time	Research province	Research district	Epidemiological method	Age (years)	Participant number	Male (N AR/ N)	Female/male (N AR/ N)	No. of patients	Event of AR (%)	Quality assessment
A 2009	Northwest China	2007.8–9	Xinjiang province	Kashgar	Random	>20	1693	/	/	231	13.64	*B*
Chen 2016	East China	2004.10–2005.10	Zhejiang province	NingBo city	Multistage sampling and cluster sampling are combined	18–70	2580	208/1281	217/1299	425	16.47	*A*
Deng 2021	North China	2019.3–10	Inner Mongolia	Chifeng, Hohhot, Erdos	Multistage stratified random sampling	16–65	5959	413/3203	501/2756	914	15.33	*A*
Huang 2018	North China	2011.11–12	Beijing	Huairou district	Stratified two-stage cluster sampling	>15	1028	68/405	99/679	158	15.37	*A*
Li 2014	South China	2009.12–2010.3	Guangdong	Guangzhou	Stratified multistage sampling	—	9899	352/5266	266/4633	618	6.2	*A*
Li 2015	North China	2013. 9–2014.1	Beijing	Chaoyang, Haidian, Shijingshan, Daxing, Shunyi, Miyun county	Stratified random cluster sampling	>20	1779	/	/	448	25.18	*A*
Ma 2020	North China	2015.5–8	Inner Mongolia	Tongliao, Jarud Banner, Kailu County, Xilinhot, Erenhot, Duolun	Multistage, stratified, clustered, and randomized sampling	>17	3600	/	/	1308	21.8	*A*
Shen 2011	Western China	2008.1–12	Western China	Chongqing, Chengdu, Nanning, Urumqi	Multistage, stratified, and cluster sampling	>19	4518/5539/3133/4772	/	/	1396/1834/982/1847	30.89/33.11/31.34/38.70	*A*
Shen 2017	Northwest China	2013.3–9	Ningxia	Ningxia	Multistage cluster sampling	21–70	4277	325/2425	359/2811	530	12.39	*A*
Tang 2008	East China	2006.10–2007.6	Zhejiang province Hunan province	Ningbo city Yongzhou	Random stratified	18–72	4729/3447	/	/	181/55	3.8/1.59	*B*
Yu 2018	Northeast China	2015	Liaoning province	—	Multistage stratified random sampling	>40	1.026	121/477	90/549	211	20.56	*A*
Zheng 2015	North China	2008.4–8	Hebei province Beijing	Xin Zhuang, Fang Zhuang	Multistage stratified random sampling	>18	803/1499	359/734	444/765	153/203	19.1/13.5	*A*

**Table 2:** Characteristics of the child morbidity studies included in the meta-analysis.

First author (year)	Geographical zone	Survey time	Research province	Research district	Epidemiological method	Age (years)	Participants number	No. of patients	Event of AR (%)	Quality assessment
Bao 2011	East China	2010.6	Shanghai	Baoshan district	Cluster random sampling survey	7–12	2313	553	3.9	*A*
Deng 2016	Central China	2011.9–2012.1	Hunan province	Changsha city	Random	3–6	2598	187	7.2	*A*
Deng 2021	North China	2019.3–10	Inner Mongolia	Chifeng, Hohhot, Erdos	Multistage stratified random sampling	6–15	266	119	44.74	*A*
Duan 2007	East China	2005. 8–12	Shandong province	Zibo city	Random	10–11	6148	228	3.7	*B*
Gao 2010	Northwest China	2009.3–9	Xinjiang province	Tianshan district, Shuimogou district, Shaybak district	Random cluster sampling	3–7	2815	622	22.1	*A*
Gao 2018	East China	2008.6	Shandong province	Zaoyang city	Cluster sampling	6–12	1290	177	13.7	*B*
Han 2009	Northwest China	2008.7	Xinjing province	Shihezi city	All primary school	9–10	2205	277	12.56	*B*
Hu 2017	Southwest China	2017.3–6	Chongqing city	_	Random cluster sampling	2–12	1170	334	28.5	*A*
Hwang 2006	Southeast China	2001	Taiwan province	_	Random stratified sampling	6–15	32143	8202	25.5	*A*
Jiang 2006	Southeast China	2004.3–9	Jiangsu province	Nanjing city	Random cluster sampling	9–10	989	48	5.1	A
Kong 2009	Southeast China	2005.11	Hubei province	Wuhan city	Random telephone interview	3–6	1211	131	10.8	A
Li 2015	North China	2013. 9–2014.1	Beijing	Chaoyang, Haidian, Shijingshan, Daxing, Shunyi, Miyun county	Stratified random cluster sampling	≤20	437	122	27.92	A
Lv 2021	South China	2019.11	Guangdong province	Guangzhou	Random cluster sampling	Grade three-Grade five	3013	697	23.1	*A*
Ma 2020	North China	2015.5–8	Inner Mongolia	Tongliao, Jarud,Banner, Kailu County, Xilinhot, Erenhot, Duolun	Multistage, stratified, clustered, and randomized	0–17	2443	650	26.6	*A*
Shen 2011	Western China	2008.1–12	Western China	Chengdu, Nanning, Urumqi	Multistage, stratified, and cluster sampling	<19	2503/900/3134	927/241/1149	37.03/26.78/36.67	*A*
Song 2015	Central China	2011.1–2012.3	Hunan province	Changsha city	Random stratified sampling survey	10–17	1275	515	42.5	*A*
Suo 2009	North China	2008.8–12	Shanxi province	Taiyuan	Random	10–11	752	170	22.6	*B*
Tang 2008	East China	2006.10–2007.6	Zhejiang province, Hunan province	Ningbo city, Yongzhou city	Random stratified	1–18	930/863	51/16	5.48/1.85	*B*
Wei 2009	South China	2008.7∼2008.12	Guangdong	Shantou	Stratified random sampling	7–16	932	157	16.8	*A*
Wu 2008	South China	2006.4–11	Guangdong	Zhuhai	Random cluster sampling	7～11	854	131	15.3	*A*
Yang 2019	Southeast China	2016.1–2018.12	Fujian province	Xiamen city	Random	6–12	1674	229	13.68	*B*
Zhang 2013	North China	2007.4–9	Beijing	Dongcheng district, Daxing district	Two-stage, clustered, and stratified random, sample study	3, 4, 5	2133/1874	997/925	53.2/43.4	*A*
Zhao 2015	Northwest China	2012.3–2013.4	Yinchuan city	Xingqing, Jinfeng, Xixia, Helan county	Random	5–14	662	97	14.65	*B*

## Data Availability

The data can be made available upon request to the corresponding author.
